The article "A Comprehensive Exploration of the lncRNA CCAT2: A Pan-Cancer Analysis Based on 33 Cancer Types and 13285 Cases" was published in 2020. Journal: Dis Markers.

# A Comprehensive Exploration of the lncRNA CCAT2: A Pan-Cancer Analysis Based on 33 Cancer Types and 13285 Cases

**DOI:** 10.1155/2020/5354702

**Published:** 2020-02-24

**Authors:** Bowen Huang, Min Yu, Renguo Guan, Dong Liu, Baohua Hou

**Affiliations:** ^1^The Second School of Clinical Medicine, Southern Medical University, Guangzhou, Guangdong Province, 510515, China; ^2^Department of General Surgery, Guangdong Provincial People's Hospital, Guangdong Academy of Medical Sciences, Guangzhou, Guangdong Province, 510080, China; ^3^Jinan University, Guangzhou, Guangdong Province, 510632, China

## Abstract

Whether the lncRNA CCAT2 expression level affects the clinical progression and outcome of cancer patients has not yet been fully elucidated. There is still an inconsistent view regarding the correlation between CCAT2 expression and clinicopathological factors, including survival data. Besides, the regulation mechanism of CCAT2 in human cancer is still unclear. Our study analyzed a large number of publication data and TCGA databases to identify the association of CCAT2 expression with clinicopathological factors and to explore the regulatory mechanisms in human cancers. We designed a comprehensive study to determine the expression of CCAT2 in human cancer by designing a meta-analysis of 20 selected studies and the TCGA database, using StataSE 12.0 to explore the relationship between CCAT2 expression and both the prognosis and clinicopathological features of 33 cancer types and 13285 tumor patients. Moreover, we performed GO and KEGG pathway enrichment analyses on potential target genes of CCAT2 collected from GEPIA and LncRNA2Target V2.0. The level of CCAT2 expression in tumor tissues is higher than that in paired normal tissues and is significantly associated with a poor prognosis in cancer patients. Besides, overexpression of CCAT2 was significantly associated with tumor size, clinical stage, and TNM classification. Meanwhile, CCAT2 expression is the highest in stage II of human cancer, followed by stage III. Finally, 111 validated target gene symbols were identified, and GO and KEGG demonstrated that the CCAT2 validation target was significantly enriched in several pathways, including microRNAs in the cancer pathway. In summary, CCAT2 can be a potential biomarker associated with the progression and prognosis of human cancer.

## 1. Introduction

The rapid advancement of exploring ncRNA is the result of RNA-Seq technology, which provides a deeper understanding of the human transcriptome. Further research on these RNAs will lead to new perspectives on cancer cell regulation mechanisms and innovative therapeutic targets [1]. According to the ncRNA length, we divided it into two categories. Short RNA has a transcript of fewer than 200 nucleotides, including miRNA, siRNA, and piRNA. Besides, transcripts longer than 200 nucleotides are classified as lncRNA [2]. NcRNA does not encode a protein, which was previously thought to be transcriptional noise or evolutionary junk [3]. However, ncRNA plays a vital role in a variety of biological processes [4]. LncRNA acts as a regulator of gene expression to regulate the development and progression of many diseases, especially malignant tumors [5, 6]. Therefore, lncRNA is used as a biomarker to monitor tumor prognosis. For example, He et al. explored the association between lncRNA PVT1 and patient prognosis in the TCGA database and sought after some possible pathways of PVT1 [7].

CCAT2 is located in the 8q24 gene desert. The locus was first named in colon tumor tissue in the 2000s [8]. The CCAT2 genomic locus, including SNP rs6983267, is associated with an increased risk of various malignancies [9]. Overexpression of CCAT2 promotes the proliferation and invasion of malignant tumors, claiming that CCAT2 plays a carcinogenic role [10]. Studies also observed that CCAT2 expression levels in tumor samples were higher than those in adjacent tissues and were associated with poor prognosis [11]. Moreover, different expression levels of CCAT2 will affect the therapeutic effects of different treatment procedures, such as chemotherapy [12].

The above evidence indicates that CCAT2 is involved in tumor progression. Moreover, some previous meta-analyses have reported that increased CCAT2 expression is significantly associated with lymph node metastasis, distant metastasis, and higher clinical stage [13, 14]. However, sample quantity is limited, and the relevance of CCAT2 to other clinicopathological parameters has not been adequately studied in these studies. Therefore, we reviewed the entire literature and searched the TCGA database for current research to explore the clinical pathology and prognostic value of CCAT2 in various types of cancer patients. We also listed potential target genes for CCAT2 by GO and KEGG analysis, and this paper discusses the possible mechanism of action of CCAT2 in tumor progression.

## 2. Material and Methods

### 2.1. Literature Review and Selection

We searched the English and Chinese medical literature in PubMed, Web of Science, Wiley Online Library, Weipu, Wangfang Data, and CNKI to identify all publications related to CCAT2 in cancer patients. The search strategy combining the terms “CCAT2” or “colon cancer associated transcript 2” is based on the purpose of the study. We also reviewed comments and references related to CCAT2 by other methods, including the extraction of previous articles cited in the meta-analysis of CCAT2 [13–15]. The deadline for our project was on December 29, 2019.

The meta-analysis study was evaluated by two independent investigators (RG Guan and D Liu) using the same multistep approach. First, check the headlines and abstracts to exclude unqualified studies that are not relevant, duplicate papers, reviews, or case reports. What is more, the full text of the remaining studies was further examined separately by the same investigator (M Yu). Finally, the third commentator (BW Huang) resolved any disputes.

We consider studies that meet the following inclusion criteria to be eligible: (i) collecting clinical samples from tumor tissue, (ii) studying the association between CCAT2 and survival data and performing CCAT2 levels by qRT-PCR quantification, and (iii) providing sufficient data to determine the HR value and its 95% CI. The exclusion criteria were as follows: (i) repeated studies, (ii) study data not sufficient to calculate HR values, (iii) studies of animals or cell lines, and (iv) reviews, comments, letters, case reports, and conference articles. If the survival analysis is not sufficient to calculate the HR value, we try to contact the author to obtain the raw survival data.

### 2.2. Data Extraction

The following relevant information from all eligible studies was extracted: first author name, publication year, country, cancer type, sample size, assay method, the criterion for dividing CCAT2 into high and low groups, follow-up time, prognostic data, age classification, gender ratio, tumor size, clinical stage, TNM classification, and histological differentiation. If the paper does not provide complete survival data, we follow the methods of He et al. [7]. The HR and 95% CI were extracted indirectly from the Kaplan-Meier survival curve using Engauge Digitizer version 11.2 (https://github.com/markummitchell/engauge-digitizer/releases).

### 2.3. Quality Assessment

The NOS was used to assess the methodological quality of two investigators (RG Guan and D Liu) independently evaluating eligible projects. They rated each study according to the following system: (i) selection, 0-4; (ii) comparability, 0-2; and (iii) exposure, 0-3. The highest score is 9 points, and score ≥ 6 indicates that the research quality is good.

### 2.4. Statistical Analysis

We used StataSE 12.0 software to analyze the information extracted from eligible studies. HR and 95% CI assessed survival data. The OR and 95% CI were calculated to analyze the relationship between human cancer and clinicopathological parameters, including age, gender, tumor size, clinical stage, TNM classification, and histological differentiation. What is more, subgroup analyses were based on the source of tumor type and overall survival data. The Cochrane *Q* test and the *I*^2^ index were used to assess potential heterogeneity in selected studies, with *P*′ < 0.05 or *I*^2^ > 50% considered statistically significant. If the selected parameter has significant heterogeneity (*P*′ < 0.05), the random effects model is used to calculate the HR value; otherwise, a fixed effects model will be employed. Finally, Begg's test was used to estimate publication bias (bilateral *P*′ < 0.05 was considered statistically significant).

### 2.5. Analysis of CCAT2 Expression Levels in All Cancers Based on TCGA Data

CCAT2 expression levels and overall survival data in the TCGA database were extracted from starBase (http://starbase.sysu.edu.cn/). Experimental data were divided into high and low groups based on the median level of CCAT2 expression. The Cox proportional hazard model of SPSS 22.0 was used to assess the effect of CCAT2 overexpression on survival. The box diagram and bar graph of CCAT2 expression in tumor samples and adjacent normal tissues were drawn by R 3.6.0 (https://www.r-project.org/) and established on the data extraction of the TCGA database (https://portal.gdc.cancer.gov/).

### 2.6. Pathway Analysis of GO and KEGG for CCAT2 Verification of Target Genes

We used GEPIA (http://gepia.cancer-pku.cn/) and LncRNA2Target V2.0 (http://123.59.132.21/lncrna2target/index.jsp) based on all published lncRNA papers to identify potential CCAT2 target genes in human cancer. GO enrichment analysis and KEGG pathway analysis were performed using DAVID Bioinformatics Resources 6.8 (https://david.ncifcrf.gov/). We used R 3.6.0 to visualize the results of GO and KEGG and used Cytoscape 3.7.1 (https://cytoscape.org/) software to display a network of CCAT2 and its related genes.

## 3. Results

### 3.1. Summary of Literature Selection and Study Characteristics

We researched to analyze the connection between CCAT2 expression and prognosis in cancer patients in all published literature (Figure 1). A total of 1304 potential studies were identified after the first search, 177 of which were considered eligible after the title and abstract screening. Next, we examined the full text of the remaining articles. Finally, 20 studies (*n* = 2192) were included in our analysis, and the main characteristics are shown in Table 1. The follow-up period was between 40 and 100 months. All selected studies investigated the relationship between CCAT2 and survival analysis, including OS, PFS, RFS, or DFS; 15 studies explored the association between CCAT2 and age, 11 for gender, 15 for tumor size, 14 for clinical stage, 6 for T classification, 12 for N classification, 7 for M classification, and 11 for histological differentiation (shown in Table 2).

### 3.2. Correlation between lncRNA CCAT2 and Clinicopathological Characteristics of the Study Patients

As shown in Table 2, we discovered that a high CCAT2 level was remarkably related to tumor size (OR = 1.50, 95% CI: 1.03-2.20, *P* = 0.036, *I*^2^ = 70.4%, and *P*′ < 0.001) (Figure 2(c)), clinical stage (OR = 3.09, 95% CI: 2.49-3.83, *P* < 0.001, *I*^2^ = 19.8%, and *P*′ = 0.238) (Figure 2(d)), T stages (OR = 2.37, 95% CI: 1.68-3.37, *P* < 0.001, *I*^2^ = 10.8%, and *P*′ = 0.347) (Figure 2(e)), N stage (OR = 3.33, 95% CI: 2.29-4.84, *P* < 0.001, *I*^2^ = 55.8%, and *P*′ = 0.009) (Figure 2(f)), and M stage (OR = 6.85, 95% Cl: 4.23-11.11, *P* < 0.001, *I*^2^ = 47.1%, and *P*′ = 0.078) (Figure 2(g)). However, no significant connection was found for age (OR = 1.04, 95% CI: 0.85-1.27, *P* = 0.714, *I*^2^ = 0.0%, and *P*′ = 0.741) (Figure 2(a)), gender (OR = 1.06, 95% CI: 0.84-1.35, *P* = 0.621, *I*^2^ = 0.0%, and *P*′ = 0.996) (Figure 2(b)), and histological differentiation (OR = 1.17, 95% Cl: 0.75-1.81, *P* = 0.484, *I*^2^ = 69.1%, and *P*′ < 0.001) (Figure 2(h)). The above results indicate that tumors with high CCAT2 levels appear to exhibit invasive biological behavior.

### 3.3. Correlation between lncRNA CCAT2 Expression and Survival Data

We analyzed the association of CCAT2 expression with OS based on the results of 20 selected studies (*n* = 2192) and the TCGA database (*n* = 11093), suggesting that CCAT2 overexpression is significantly associated with poor prognosis for certain cancer types. Considering the significant heterogeneity in the study, we performed two subgroup analyses based on survival data and the source of the cancer type. In a subgroup analysis of OS, we found that high expression of CCAT2 was significantly associated with poor OS in all databases (HR = 1.15, 95% CI: 1.04-1.26, *P* < 0.001), including publications (HR = 1.75, 95% CI: 1.50-2.01, *P* < 0.001) and TCGA (HR = 1.01, 95% CI: 0.90-1.12, *P* < 0.001) (Figure 3(a)). As pituitary adenoma, colorectal cancer, renal cell carcinoma, oral cancer, small cell lung cancer, ovarian cancer, prostate cancer, and esophageal cancer were studied separately, we have classified them as others. Similar results were generated in a subgroup analysis based on tumor type (hepatocellular carcinoma (HR = 2.44, 95% CI: 1.56-3.33, *P* < 0.001), osteosarcoma (HR = 1.17, 95% CI: 0.70-1.65, *P* < 0.001), cholangiocarcinoma (HR = 2.96, 95% CI: 1.95-3.97, *P* < 0.001), gastric cancer (HR = 1.47, 95% CI: 1.04-1.89, *P* < 0.001), breast cancer (HR = 1.98, 95% CI: 1.36-2.60, *P* < 0.001), and others (HR = 1.67, 95% CI: 1.40-1.94, *P* < 0.001)) (Figure 3(b)). No significant heterogeneity was found in these studies.

### 3.4. Publishing Bias

Begg's funnel plot was used to assess publication bias in our study. No publication bias was observed in studies evaluating the association of CCAT2 with clinicopathological features and OS in the study group (*P* = 0.496) and TCGA (*P* = 0.455) (Figures 4(a) and 4(b)). Similarly, we conducted a publication bias analysis on the influencing factors of OS in patients (Figures 4(c)–4(j)). Among them, suspicious publication bias was found in the tumor size subgroup (Pr = 0.038). Therefore, we used the trim method for further verification. The results indicated that the tumor size subgroup needed to increase three experiments to eliminate the bias, but the 95% CI after clipping and supplementation showed no statistical significance, reminding us that the previous results were stable.

### 3.5. The Expression Level of CCAT2 in Pan-Cancer

Based on the results obtained from TCGA, we plotted a box diagram of the CCAT2 expression profile for tumor samples and adjacent normal tissues (Figure 5(a)). We found that CCAT2 is highly expressed in 6 of 33 tumor tissues (COAD/KIRC/STAD/PRAD/ESCA/READ) (Figure 5(b)) and is weakly expressed in 4 tumor tissues (BRCA/LUSC/THCA/PAAD) (Figure 5(c)). And CCAT2 is mainly expressed in stage II of tumor pathology, followed by stage III (from GEPIA, Figure 5(d)).

### 3.6. Functional Analysis of CCAT2-Related Genes in Human Tumors

To explore the underlying mechanism of action of CCAT2, we identified a total of 111 target genes using GEPIA and LncRNA2Target V2.0. GO and KEGG analysis was performed. CCAT2 and target gene symbols were analyzed by GO enrichment analysis, including BP, CC, and MF, and the results are shown in Figure 6. Furthermore, KEGG enrichment analysis revealed that CCAT2 might play a role in cancers such as microRNAs in cancer pathway, Hippo signaling pathway, RNA degradation pathway, ribosome biogenesis in eukaryote pathway, and cell cycle pathway (Figures 6 and 7).

## 4. Discussion

Numerous studies have shown that overexpression of CCAT2 is significantly associated with clinical outcomes and other clinicopathological parameters in cancer patients [16–18]. The review article also summarizes the critical role that CCAT2 may play in the development of multiple cancers [19]. A meta-analysis also showed that the upregulation of CCAT2 was associated with lymph node metastasis, distant metastasis, and poor OS in patients with malignancy, although the association between CCAT2 and other clinicopathological parameters was not discussed in previous studies [15]. To obtain more convincing conclusions and explore the potential mechanism of action of CCAT2 in tumors, we performed current studies by combining the results of published studies with TCGA survival data followed by GO and KEGG analysis.

A meta-analysis of 2192 patients from 20 eligible studies and 11093 patients from TCGA currently explores the association between CCAT2 overexpression and prognosis, as well as the clinicopathological parameters of cancer patients. Therefore, our research is by far the most comprehensive analysis. We assessed the quality of all selected studies through NOS and used Begg's method to examine publication bias. Our results show that high expression of CCAT2 is associated with poor OS. For clinicopathological features of cancer patients, our study suggests that high CCAT2 is significantly associated with cancer growth and metastasis, including tumor size, clinical stage, and TNM classification, although age, gender, and histological differentiation are not significant factors. The results suggest that CCAT2 may be a potential tumor biomarker and is associated with tumor invasiveness, which is why CCAT2 is mainly expressed in stage II, followed by stage III.

Furthermore, a subgroup analysis of CCAT2 expression and overall survival was not statistically significant in TCGA, and CCAT2 is likely overexpressed in certain types of tumors. Besides, subgroup analysis was also performed on specific cancers, including hepatocellular carcinoma, osteosarcoma, cholangiocarcinoma, gastric carcinoma, and breast cancer. Increased CCAT2 expression was associated with worse HR observed in hepatocellular carcinoma, cholangiocarcinoma, gastric cancer, and breast cancer, whereas no significant association between CCAT2 expression and HR was detected in osteosarcoma. However, KIRC, PRAD, READ, SKCM, and STAD in the TCGA data set are associated with a good prognosis. We reviewed related studies and found that overexpression of CCAT2 levels is associated with worse outcomes in renal cell carcinoma [20], prostate cancer [21], gastric cancer [17, 22, 23], and colorectal cancer [24], and there is no corresponding melanoma report. Sampling errors and publication bias may cause the inconsistent conclusions of literature studies and TCGA in these tumors. Based on the evidence from our study, all of these results suggest that CCAT2 may serve as a reliable independent diagnostic and prognostic biomarker, and even all types of cancers with high CCAT2 expression may have a poor prognosis and more adverse clinical pathology parameters. Although these findings suggest that CCAT2 may play a role in cancer, the exact mechanism remains to be elucidated. The association between CCAT2 and the prognosis of different types of tumors needs to be confirmed with more research.

Studies have shown that CCAT2 expression levels are upregulated in cancerous tissues compared to paired adjacent tissues; the same results were found in in vitro cell line samples [25]. Research on the mechanism of action of CCAT2 in cancer has proliferated in recent years, and there is increasing evidence that CCAT2 can affect the different biological behaviors of different types of tumors. Yu et al. observed that CCAT2 could positively regulate the expression of the POU5F1B gene by inhibiting the PI3K/mTOR signaling pathway. The silencing of the CCAT2 gene inhibits the proliferation of BGC-823 cells and induces apoptosis and autophagy in BGC-823 cells [26]. Cai et al. revealed that the silencing of CCAT2 inhibited the proliferation and invasion of PANC-1 cells in vitro and reduced the tumorigenesis of PANC-1 xenografts in vivo, and KRAS regulated CCAT2 via the MEK/ERK signaling pathway [27]. Even though we have made progress in understanding the role of CCAT2 in malignant tumors, the precise molecular mechanism of its biological function remains unclear. Therefore, we collected validated CCAT2 targeting genes using the GEPIA and LncRNA2Target platforms and performed a comprehensive target gene network analysis.

The analysis of GO and KEGG pathways suggests that CCAT2 may play a key role in human tumors through different pathways, including miRNAs in the cancer pathway, etc. miRNAs are defined as small noncoding sets of 19 to 24 nucleotides associated with mRNA expression and regulate the expression of downstream gene targets, including oncogenes, tumor suppressor genes, and transcription factors [28]. Studies have shown that miRNAs are expressed in several malignancies, including hepatocellular carcinoma [29], hepatoblastoma [30], cervical cancer [31], and colon cancer [32], which play the vital part in the diagnosis and prognosis.

Compared to previous meta-analyses, our research has several advantages [13–15]. First of all, the included studies and cases extended from 11 studies with 1335 cases [13] to 20 studies and TCGA database with 13285 cases. Moreover, we performed several subgroup analyses to further explore the role of CCAT2 in different types of tumors and also achieved a significant correlation between high CCAT2 expression and worse OS in survival curve studies. Last but not least, all types of tumors were included in our study, which was lacking in previous meta-analyses. More importantly, our study found that CCAT2 is involved in tumor progression by modulating miRNAs in the cancer pathway. These findings are following previous publications that CCAT2 increases the growth, invasion, and migration of colon cancer cells and endometrial cancer cells by lncRNA-miRNA crosstalk [33, 34].

Although our study attempts to fully elucidate the association between CCAT2 and cancer progression and prognosis, our research has some limitations. For the meta-analysis, different definitions of high CCAT2 expression levels in selected studies are factors that contribute to publication bias. Besides, the current eligible countries in the meta-analysis are only China, the USA, and Japan, and more trials in other countries should confirm our research. At the same time, since there is no direct data for multivariate analysis in some existing studies, we have to extract relevant data through Kaplan-Meier curves, which may lead to deviations in HR values. More importantly, all available studies are retrospective studies that tend to be published when positive results are confirmed. Thus, the impact of CCAT2 on the prognosis and clinicopathological parameters of malignant tumors may be overestimated. Therefore, further research is needed to study the clinical significance and diagnostic value of CCAT2 in human cancer. Furthermore, although CCAT2 can act through a variety of mechanisms, based on the correlation of gene expression levels between CCAT2 and miRNA, only one possible mechanism of the role of CCAT2 in gene regulation has been investigated. In order to understand more features of CCAT2, further research is needed to explore other possible mechanisms.

In light of our findings, we believe that the expression of CCAT2 may serve as potential candidates for prognostic factors as well as therapeutic targets in malignant tumors. Of note, the prognostic roles of CCAT2 varied greatly across cancers, which implied a noteworthy amount of heterogeneity between different types of tumors. In addition, the expression of CCAT2 was closely associated with tumor size, clinical stage, and TNM classification and mainly expressed in stage II, which indicated that CCAT2 is a significant biomarker to monitor tumor progression. Current findings enhance our understanding of the CCAT2 in cancer monitor and identify strategies for the early invention in clinical management. Moreover, further illumination of the underlying mechanism and the interaction between CCAT2 and tumors may provide important implications for the success of early monitoring and prognosis prediction in cancers.

## 5. Conclusions

Our study demonstrated that a higher CCAT2 expression was significantly associated with an aggressive disease course in patients with cancer, predicting a larger tumor size, more advanced clinical stage, more inferior TNM classification, and shorter OS. We also demonstrated that CCAT2 plays an essential role in the biological processes of tumor progression via a variety of pathways.

## Figures and Tables

**Figure 1:** Flow diagram of the search and selection of study patients.

**Figure 2:** Meta-analysis estimating the correlation between CCAT2 and clinicopathological parameters in cancer patients: (a) Age (*P*′ = 0.741, fixed effects model); (b) gender (*P*′ = 0.996, fixed effects model); (c) tumor size (*P*′ < 0.001, random effects model); (d) clinical stage (*P*′ = 0.238, fixed effects model); (e) T (*P*′ = 0.347, fixed effects model); (f) N (*P*′ = 0.009, random effects model); (g) M (*P*′ = 0.078, fixed effects model); (h) differentiation (*P*′ < 0.001, random effects model).

**Figure 3:** Subgroup analyses. (a) A meta-analysis of the selected studies and TCGA data estimating the association of CCAT2 with the patients' OS (*I*^2^ ≥ 50%, random effects model). (b) Subgroup analyses of the OS based on the tumor type (*I*^2^ < 50%, fixed effects model).

**Figure 4:** Funnel plots (Begg's method) of potential publication bias in the selected studies. (a) OS of study patients (Pr = 0.496); (b) OS in TCGA data (Pr = 0.455); (c) age (Pr = 0.921); (d) gender (Pr = 1.000); (e) tumor size (Pr = 0.038); (f) clinical stage (Pr = 0.050); (g) T (Pr = 1.000); (h) N (Pr = 0.837); (i) M (Pr = 0.548); (j) differentiation (Pr = 0.213).

**Figure 5:** CCAT2 expression profile across tumor samples and adjacent normal tissues from TCGA; log_2_(TPM + 1) scale. (a) The level of CCAT2 expression of all types of tumors is shown, box plot. (b) The level of CCAT2 expression was higher in the tumor than in adjacent normal tissue (COAD/KIRC/STAD/PRAD/ESCA/READ), bar plot. (c) The level of CCAT2 expression was lower in the tumor than in adjacent normal tissue (BRCA/LUSC/THCA/PAAD), bar plot. (d) The pathological stage plot of CCAT2 from GEPIA. ^∗^The height of the bar represents the median expression of specific tumor types or normal tissues.

**Figure 6:** Bubble plot for GO/KEGG term analysis of CCAT2: (a) BPs; (b) CCs; (c) MFs; (d) KEGG pathway.

**Figure 7:** The network for the GO/KEGG analysis of CCAT2.

**Table 1:** Main characteristics of the selected studies.

First author	Year	Country	Cancer type	*N* (M/F)	High expression	Follow-up (months)	Outcome	HR (95% CI)	Quality score
Fu [35]	2019	China	HCC	122 (79/43)	>Median expression	60^∗^	OS	2.126 (1.273-8.775)	8
Ruan [36]	2018	China	OS	50 (32/18)	>Median expression	70^∗^	OS	1.32 (0.88-1.97)	8
Yan [10]	2018	China	OS	40	NR	60^∗^	OS/PFS	0.69 (0.22-2.21)/1.42 (0.55-3.62)	7
Xu [37]	2018	China	CCA	60 (27/33)	Median value: 2.95-fold	60^∗^	OS	2.391 (1.024-5.583)	8
Fu [38]	2018	China	PA	74	>Median expression	40^∗^	OS	1.56 (1.06-2.29)	7
Bai [39]	2018	China	CCA	106 (78/28)	Above the cut-off value	72^∗^	OS/PFS	3.10 (2.17-4.43)/3.31 (2.32-4.72)	8
Chen [40]	2017	China	HCC	60 (48/12)	>Median expression	40^∗^	OS	2.46 (1.71-3.53)	8
Ozawa [24]	2017	USA/Japan	CRC	300	NR	60^∗^	OS/RFS	2.40 (1.22-4.59)/2.39 (1.10-5.08)	7
Wu [22]	2017	China	GC	208 (124/84)	>twofold change	85	OS/DFS	1.214 (0.898-1.882)/1.687 (0.833-1.896)	8
Huang [20]	2017	China	RCC	61 (34/27)	>Median expression	60^∗^	OS	3.02 (1.14-7.96)	8
Ma [41]	2017	China	OC	62 (40/22)	>eightfold	60^∗^	OS	1.60 (1.03-2.47)	8
Deng [42]	2017	China	BC	120	>Median expression	100^∗^	OS	1.89 (1.36-2.63)	8
Chen [18]	2016	China	SCLC	112 (67 : 45)	>Median expression	60^∗^	OS	1.66 (1.22-2.27)	7
Wang [23]	2016	China	GC	108 (64 : 44)	>Median expression	70^∗^	OS/DFS	2.108 (1.442-3.202)/2.305 (1.554-3.418)	8
Huang [43]	2016	China	ORC	109	>Median expression	60^∗^	OS/DFS	2.938 (1.526-5.873)/1.74 (1.27-2.39)	8
Zheng [21]	2016	China	PC	96	>Median expression	60^∗^	OS/PFS	2.292 (1.370-3.528)/2.276 (1.199-2.768)	7
Zhang [16]	2015	China	EC	229 (170/59)	>Median expression	80^∗^	OS	1.432 (1.005-2.041)	8
Wang [17]	2015	China	GC	85 (41/44)	>Mean expression	60^∗^	OS/PFS	2.405 (1.194-5.417)/2.315 (1.097-5.283)	8
Cai [44]	2015	China	BC	67	>eightfold	60^∗^	OS	3.57 (1.77-7.21)	7
Chen [45]	2015	China	CC	123	>Mean expression	60^∗^	OS/PFS	2.813 (1.504-6.172)/3.072 (1.716-8.174)	8

*N* (M/F): number (male/female); HR: hazard ratio; CI: confidence interval; HCC: hepatocellular carcinoma; OS: osteosarcoma; CCA: cholangiocarcinoma; PA: pituitary adenomas; CRC: colorectal carcinoma; GC: gastric carcinoma; RCC: renal cell carcinoma; OC: oral carcinoma; BC: breast cancer; SCLC: small cell lung cancer; ORC: ovarian cancer; PC: prostate cancer; EC: esophageal carcinoma; CC: cervical cancer; OS: overall survival; PFS: progression-free survival; RFS: relapse-free survival; DFS: disease-free survival; NR: not reported; ^∗^Approximate times extracted from survival curve.

**Table 2:** Combinations of data evaluating the associations of CCAT2 with the clinicopathological characteristics of the study patients.

Clinicopathological parameters	Studies (*n*)	Test/event total		Control/event total		Model	OR (95% CI)	Test for heterogeneity		*P* value
								*I* ^2^	*P*′	
Age (old/young)	15 (1649)	449	859	405	790	Fixed	1.04 (0.85-1.27)	0.0%	0.741	0.714
Gender (male/female)	11 (1201)	392	764	221	437	Fixed	1.06 (0.84-1.35)	0.0%	0.996	0.621
Tumor size (large/small)	15 (1656)	418	761	435	895	Random	1.50 (1.03-2.20)	70.4%	0.000	0.036
Clinical stage (advanced/early)	14 (1584)	568	891	258	693	Fixed	3.09 (2.49-3.83)	19.8%	0.238	0.000
T (T3-T4/T1-T2)	6 (579)	145	231	147	348	Fixed	2.37 (1.68-3.37)	10.8%	0.347	0.000
N (N1-N3/N0)	12 (1356)	399	602	306	754	Random	3.33 (2.29-4.84)	55.8%	0.009	0.000
M (M1/M0)	7 (690)	118	142	224	548	Fixed	6.85 (4.23-11.11)	47.1%	0.078	0.000
Differentiation (poorly/well)	11 (1331)	324	616	349	715	Random	1.17 (0.75-1.81)	69.1%	0.000	0.484

## Data Availability

Data from cancer patients used in this study were collected in the published papers and the TCGA database. The results of the statistical analysis of these data were placed in this manuscript.

## Abbreviations

lncRNA: Long noncoding RNA
CCAT2: Colon cancer-associated transcript 2 gene
TCGA: The Cancer Genome Atlas
GO: Gene Ontology
KEGG: Kyoto Encyclopedia of Genes and Genomes
T: Tumor classification
N: Lymph node classification
M: Metastasis classification
ncRNA: Noncoding RNA
RNA-Seq: RNA deep sequencing
CNKI: China National Knowledge Infrastructure
qRT-PCR: Quantitative real-time polymerase chain reaction
NOS: Newcastle-Ottawa Scale
HR: Hazard ratio
CI: Confidence interval
OR: Odds ratio
OS: Overall survival
PFS: Progression-free survival
RFS: Recurrence-free survival
DFS: Disease-free survival
miRNA: MicroRNA
BP: Biological processes
CC: Cellular components
MF: Molecular factors.
